# Computed Tomography Image Features under Convolutional Neural Network Algorithm in Analysis of Inflammatory Factor Level and Prognosis of Patients with Hepatitis B Virus-Associated Acute-on-Chronic Liver Failure

**DOI:** 10.1155/2021/2110612

**Published:** 2021-11-08

**Authors:** Zhibing Xie, Li Ding, Yongzhong Li

**Affiliations:** ^1^Infectious Disease Center, Huaihua First People's Hospital, Huaihua 418000, Hunan, China; ^2^Breast and Thyroid Surgery, Huaihua First People's Hospital, Huaihua 418000, Hunan, China

## Abstract

This study aimed to explore the application value of three-dimensional (3D) convolutional neural networks (3D-CNN)-based computed tomography (CT) image intelligent segmentation model in the identification of lesions of patients with hepatitis B virus-associated acute-on-chronic liver failure (HBV-ACLF). A total of 30 patients with HBV-ACLF, 30 patients with chronic HBV hospitalized in hospital, and 30 healthy volunteers were selected as subjects. Liver function and serum inflammatory factors were measured in each group, and the 3D-CNN algorithm model was applied to CT imaging. The results showed that the levels of interleukin (IL)-6, IL-26, and IL-37 in the HBV-ACLF group were the highest, which were 128.43 ± 45.16 pg/mL, 1237.47 ± 536.22 pg/mL, and 50.83 ± 7.62 pg/mL, respectively. Total bilirubin (TBIL) (*P*=0.035) and IL-26 (*P*=0.013) were independent predictors that affected the prognosis of HBV-ACLF patients. The results of lesion segmentation showed that the Dice coefficient of 3D-CNN low-density focus and enhanced focus segmentation was the highest (0.821 ± 0.07 and 0.773 ± 0.071), and the marked area was close to the area manually drawn by the doctor. 3D CNN was superior to other algorithms in the number of nodular lesions detected (533), sensitivity (97.5%), and missed detection rate (0.52%) (*P* < 0.05). In short, IL-26 may become a useful biomarker in the treatment of HBV-ACLF. The 3D-CNN model improved the segmentation performance of lesions in CT images of HBV-ACLF patients, which provided a reference for the diagnosis and prognosis of HBV-ACLF.

## 1. Introduction

Acute-on-chronic liver failure (ACLF) refers to the acute deterioration of liver failure syndrome in patients with chronic liver disease whose liver function is originally stable under the action of various acute injury factors [1, 2]. Related research pointed out that more than 30% of ACLF patients are caused by infection, and the main cause of ACLF in China is hepatitis B virus (HBV) infection [3]. The patient's infection index has risen greatly, which is directly proportional to the severity of the disease and the mortality rate. This type of infection is mainly caused by bacteria such as Gram-negative bacilli. However, in recent years, with the abuse of antibiotics and the increase in the types of multidrug resistant bacteria, the infection range of HBV-ACLF patients is gradually expanding [4]. Bacteria generally induce inflammation through pathogen-associated molecular patterns (PAMPs) and virulent factors [5]. Studies found that the possible involvement in the pathogenesis of HBV-ACLF includes immune damage, inflammation, and cell apoptosis. It shows that the level of inflammatory factors in serum will change when HBV-ACLF occurs [6, 7], and its expression has potential clinical treatment and prognostic evaluation value.

Image omics is a technology that deeply mines data features from medical images through high-throughput multidimensional analysis [8]. The use of advanced image analysis tools and various data statistics and analysis tools for accurate diagnosis provides a powerful tool for modern medicine [9, 10]. In recent years, with the development of big data and medical imaging, imaging omics has been widely used in the prediction of the internal microscopic manifestations, pathological manifestations, and gene expression of clinical lesions [11]. Among them, computed tomography (CT) is the most valuable examination method at present. CT plain scan can describe the morphological characteristics of the lesion and clarify the status of the lesion, while the enhanced CT scan can reflect the characteristics of the blood supply of the lesion and the relationship with the surrounding tissue structure [12]. However, it is not ideal for the segmentation of low-density or nodular lesions in the liver of HBV-associated ACLF patients. CT images have many slices, and the size, location, and shape of low-density lesions are inconsistent. Manual reading is time-consuming and laborious, and there is no uniform standard for segmentation results. It is easy to have inconsistent diagnosis results from different doctors [13, 14]. Therefore, more intelligent algorithms are needed for image segmentation.

Convolutional neural network (CNN) has demonstrated more substantial effects and better clinical application prospects than traditional shallow learning methods in image segmentation and classification [15]. However, most of them are based on 2D cross section for feature extraction, and it is difficult to make full use of the data correlation in the vertical axis [16]. On this basis, an automatic segmentation algorithm based on 3D CNN for dual-channel 3D dense connection network is proposed. Convolution kernels of different sizes are used to extract multiscale features under different scale receptive fields. Then, the densely connected blocks of each channel were used for feature learning and transmission. After the features were connected, they were input to the classification layer to classify the target volume element [17, 18], and finally the automatic segmentation of the lesion was realized.

To sum up, the use of 3D-CNN model to optimize medical CT images to assist physicians in detecting low-density foci or nodular lesions in the liver of patients with HBV-associated ACLF has become a hot topic of current research by scholars. In this study, liver function and serum inflammatory cytokine levels were detected in 30 HBV-associated ACLF patients, 30 CHB patients, and 30 healthy volunteers. The end-to-end neural network architecture was designed based on 3D-CNN and applied to CT image analysis, to comprehensively evaluate the application value of 3D-CNN algorithm combined with CT imaging in the level of inflammatory factors and prognosis of HBV-associated ACLF patients.

## 2. Materials and Methods

### 2.1. Research Objects

A total of 30 patients with HBV-associated ACLF hospitalized in hospital from May 2019 to May 2020 were collected, with an age range of 30–80 years. Chronic active hepatitis B (CHB) patients were 30 cases, aged 31–77 years. Thirty healthy volunteers who underwent physical examination in this hospital during the same period were selected as healthy control group, aged 20–67 years.

Inclusion criteria for HBV-associated ACLF were as follows: patients who were in line with the diagnostic criteria of Guidelines for Diagnosis and Treatment of Liver Failure published by Liver Failure and Artificial Liver Research Group of Chinese Association of Infectious Diseases in 2018 [19] and serum total bilirubin in patients being 10 times or more than the normal value or increased by 17.1 *μ*mol/L/day. Exclusion criteria were as follows: patients who had coinfection with other hepatitis viruses or immunodeficiency viruses, patients with drug-induced hepatitis and alcoholic liver, patients who had liver disease caused by parasitic infection, patients with hyperthyroidism, women in pregnancy or lactating period, and patients with liver metastasis of primary liver cancer or malignant tumor.

Inclusion criteria for CHB patients were the following: patients who were in line with the diagnostic criteria of Guidelines for Prevention and Treatment of chronic hepatitis B published by the Chinese Society of Liver Diseases and the Chinese Society of Infectious Diseases in 2015 [20] and the history of infection being more than six months. Exclusion criteria were the following: patients complicated with other viral hepatitis; patients with alcoholic liver, cirrhosis, drug-induced hepatitis, or fatty liver; patients with genetic metabolic liver disease; patients with autoimmune liver disease or parasitic liver disease; and patients with liver metastasis of primary liver cancer or malignant tumor.

Inclusion criteria of healthy volunteers were the following: all examination indexes and biochemical indexes being normal, and the patients not taking any drugs in the past week. Exclusion criteria were the following: those with organic diseases.

This experiment had been approved by the ethics committee of the hospital. All the experimental matters had been informed to the subjects and their families, who had signed informed consent.

### 2.2. Main Instruments and Reagents

Automatic blood coagulation analyzer was from Nanjing VEDENG Medical Co., Ltd. Centrifuge was from Nanjing Yiruoda Instrument Equipment Co., Ltd. Low-temperature refrigerator was from Jinan OLABO Instrument Equipment Co., Ltd. Microplate reader was from Jinan Laobao Medical Equipment Co., Ltd. Interleukin- (IL-) 26 kit was from Shanghai Yiyan Biotechnology Co., Ltd. IL-6 kit was from Shanghai Tongwei Industrial Co., Ltd. IL-27 kit was from Shanghai Jichun Industrial Co., Ltd. Enzyme conjugate was from Shanghai Rayzbio Biotechnology Co., Ltd. Termination fluid was from Shanghai Acmec Biochemical Co., Ltd.

### 2.3. Liver Function and Inflammatory Factor Detection

5 mL of fasting venous blood was collected from all participants in the morning. After the blood sample was coagulated, it was centrifuged at a frequency of 3,500 rpm for 10 minutes. If the sample did not show hemolysis or lipemia, the upper serum was taken and stored in a refrigerator at −80°C. Routine detections were implemented for alanine aminotransferase (ALT), aspartate aminotransferase (AST), serum total bilirubin (TBIL), prothrombin time (PT), and activated partial thromboplastin time (APTT) using automatic serum coagulation analyzer. IL-26 was measured by double-antibody sandwich enzyme-linked immunosorbent assay (ELISA). The kit was taken out from the 4°C refrigerator and cooled to room temperature. The distilled water was diluted in a ratio of 1 : 20, and washing solution was prepared. The standard material was diluted to different concentrations, and 100 *μ*L of the tested serum sample was injected into the well of the ELISA plate. The plate was sealed and left standing at 37°C for 1 hour; then, the plate was thoroughly cleaned for five times and dried. 100 *μ*L biotinylated antibody was injected into each well, and the sealed plates were stood at 37°C for 1 hour. The plate was cleaned five times and dried. 100 *μ*L enzymatic conjugate was added into each well, standing at 37°C for 15 min. The plate was cleaned five times and dried. Then, 50 *μ*L of substrates A and B was added into each well, standing for 15 minutes at 37°C in dark. One drop of terminating solution was added to each well to terminate the experimental reaction. The absorbance was measured at 450 nm using a microplate analyzer. The operation for the determination of IL-6 and IL-27 was the same as above.

### 2.4. CNN Algorithm

Convolutional network is a kind of neural network structure, which is regarded as a special artificial neural network. The input data is calculated through the multilayer nonlinear mapping, and the prediction result is output. Its essence is a regression optimization calculation, which introduces a feedback layer into the traditional multilayer perception network structure to optimize the prediction results. It mixes A convolutional layer-activation layer, extracts image feature information, connects a pooling layer for downsampling, and repeats it many times until the image is minimized. Then, it connects a fully connected layer to convert all feature images into feature vectors. Finally, the result is obtained through the output layer. The basic network structure is shown in Figure 1.

The convolutional layer extracts the feature information of a certain area, and the image obtained after convolution is the feature map. In the CNN, the convolutional layer has two key characteristics of local connection and weight sharing. The meaning of local connection is that each point in the back layer only connects the corresponding area in the front layer. Weight sharing means that it inputs a picture and scans it with a convolution kernel. The number in the convolution kernel is called the weight. Each position in this picture is scanned by the same convolution kernel, so the weight is the same; that is, it is shared. The structure diagram is roughly as shown in Figure 2.

In the CNN, the definition of the 3D convolutional layer is as follows:

(1) $$\begin{array}{c} I_{n}^{j}\left(a,b,c\right)=\sum_{h}\sum_{e,f,g}I_{h}^{j-1}\left(a-e,b-f,c-g\right)M_{\mathrm{hn}}^{j}\left(e,f,g\right)+p_{n}^{j}. \end{array}$$

Here, *I*_*n*_^*j*^ ∈ *θ*^3^ is the *n*th feature image representing the *j*th layer, *M*_hn_^*j*^ ∈ *θ*^3^ is the 3D convolution kernel connecting *I*_*h*_^*j*−1^ and *I*_*n*_^*j*^, and *p*_*n*_^*j*^ ∈ *θ*^3^ is the offset of connecting _*I*_^*j*−1^ and *I*_*n*_^*j*^. A convolution kernel moves in the layer of the neural network, thereby obtaining a feature image of the next layer. The expression of the size of the image is as follows:

(2) $$\begin{array}{c} O_{\mathrm{out}}=\frac{O_{\mathrm{in}}-Q+2R}{T}+1. \end{array}$$

Here, *O*_in_ is the size of the input feature image, *Q* is the size of the corresponding convolution kernel, *R* is the number of boundary zero padding, and *T* represents the length of the convolution kernel when it moves. In the neural network, there are two main types of pooling layers, the largest pool and the average pool. The calculation method of the maximum pool is as follows:

(3) $$\begin{array}{c} I_{n}^{j}\left(a,b,c\right)=\underset{0\leq e,f,g\leq w}{\max}\left\{I_{n}^{j-1}\left(a\cdot w+e,b\cdot w+f,c\cdot w+g\right)\right\}. \end{array}$$

The average pool is expressed as follows:

(4) $$\begin{array}{c} I_{n}^{j}\left(a,b,c\right)=\frac{1}{w^{3}}\sum_{e=0}^{w}\sum_{f=0}^{w}\sum_{g=0}^{w}I_{n}^{j-1}\left(a\cdot w+e,b\cdot w+f,c\cdot w+g\right). \end{array}$$

Here, *w* is the size of pooling. After passing through the pooling layer, the number of feature maps does not change, and the size of the image is calculated by the following equation:

(5) $$\begin{array}{c} O_{\mathrm{out}}=\frac{O_{\mathrm{in}}-w}{T}+1. \end{array}$$

Here, *O*_in_ is the size of the input feature image, *w* is the pooling size, and *T* is the pooling step size. For the fully connected layer, each neuron in it will be connected to the previous layer, and the Softmax layer is often used as the output layer of the CNN. Its expression is as follows:

(6) $$\begin{array}{c} I_{u}^{N}=\frac{x^{I_{u}^{N-1}}}{\sum {}_{v=1}^{v}x^{I_{v}^{N-1}}}\mathrm{for}\;u=1,\cdots ,V. \end{array}$$

Here, *V* represents the total number of categories, *N* is the total number of layers of the neural network, *I*_*V*_^*N*−1^ is the *v* th node in the *N* − 1 th layer (usually a fully connected layer), and *I*_*u*_^*N*^ represents the *u*th node in the *N*th layer (i.e., the output layer). The sum of the probabilities of all categories is 1.

Since most of the low-density areas of the liver occupy a small area in the image, the channels in the network are usually used to sample under the pooling layer to avoid excessive loss of small information. The convolution module is employed to extract the information of this layer, and then deconvolution is performed to generate cascade with the feature image, which enables multilevel feature learning, thereby helping to detect low-density areas of different sizes.

### 2.5. 3D-CNN

2D-CNNs mainly focus on 2D neighborhood information, while 3D-CNN is calculated through three dimensions and extracts features in 3D space. The main content of this study is applying 3D-CNN to the segmentation of low-density lesions in the liver area.

CNNs are individually estimated according to the neighborhood and context of each volume element in the image, and feature extraction is completed by cascading a series of convolution operations. 3D-CNN uses a 3D convolution kernel, facing the initial 3D data, which completes the convolution calculation through the input layer and the convolution kernel. After addition of the bias term, the nonlinear excitation function is used to obtain the output characteristic image. The basic network structure is shown in Figure 3.

The calculation method is expressed as follows:

(7) $$\begin{array}{c} y_{z-1}^{u}=g\left(\sum q_{z}^{u,v}⊗y_{z-1}^{v}+d_{z}^{u}\right). \end{array}$$

Here, each *q*_*z*_^*u*,*v*^ is the learned hidden weight, *u* represents the number of convolution kernels (the dimension of the output feature), *v* represents the dimension of the input feature, *y*_*z*−1_^*v*^ represents the output 3D feature map, *d*_*z*_^*u*^ represents the bias term, ⊗ is the convolution calculation, and *g* represents the nonlinear activation function. In 3D-CNN, if features are input to the network layer with a higher level, complex features will appear, which are used for classification. The end of the CNN is the classification layer, which is compared with the labels used for classification. This layer generally uses a normalized exponential function, which is defined and expressed as follows:

(8) $$\begin{array}{c} x_{s}=\frac{r^{O_{s}}}{\sum_{s}^{N}r^{O_{s}}}. \end{array}$$

Here, *O*_*s*_ represents the output of the previous layer, *s* represents the index number of the estimated category, *N* is the number of categories in the layer, and *x*_*s*_ represents the ratio of the index of the estimated category at this time to the sum of all category factors. With the help of Softmax, the output value of each category is adjusted to the estimated probability compared with it.

### 2.6. Low-Density Foci Segmentation Based on 3D-CNN

The low-density stove segmentation process based on 3D-CNN is shown in Figure 4. In the training stage, the training set image is input, and the volume elements are normalized through preprocessing. Then, the features of each dimension are learned and extracted. According to the estimated conclusion and classification label, the patches generated by the loss function in the training and test set images are counted and then normalized. The categories of the volume elements are calculated through the network model one by one, and the segmentation result image is output.

### 2.7. CT Examination

A Brilliance 64-row helical scanner (GE Company, USA) was employed for inspection. The layer thickness was 5 mm, the spacing was 5 mm, and the reconstruction layer thickness was 0.625 mm. The tube current was 380 mA, the tube voltage was 125 kV, and the collimator width was 0.625 mm. In the enhanced scan, 80–100 mL (350 mg/100 mL) of the contrast agent iohexol was injected at a flow rate of 3-4 mL/s. Scanning phases were 20–25 s in the arterial phase, 65–70 s in the venous phase, and 180 s in the delayed phase. The image data was processed by the system's own imaging workstation.

### 2.8. Statistical Analysis

SPSS 24.0 was used for statistical analysis of all experimental data. The continuous variables conforming to normal distribution were represented as mean ± standard deviation ($\bar{\text{x}}$ ± *s*), and the *t*-test was used for comparison between groups. One-way analysis of variance was used for comparison between multiple groups. Multivariate analysis was performed using logistic regression equation analysis. The correlation was assessed by Pearson test. *P* < 0.05 was considered statistically considerable.

## 3. Results

### 3.1. Comparison of the Levels of Inflammatory Factors among the Three Groups of Objects

In Figure 5, IL-6, IL-26, and IL-37 in the HBV-ACLF group were 128.43 ± 45.16 pg/mL, 1237.47 ± 536.22 pg/mL, and 50.83 ± 7.62 pg/mL, respectively, which were higher than those of 89.17 ± 28.39 pg/mL, 689.14 ± 351.7 pg/mL, and 31.19 ± 5.82 pg/mL in CHB group and those of the healthy group 58.45 ± 13.22 pg/mL, 116.43 ± 56.29 pg/mL, and 14.14 ± 2.18 pg/mL, respectively. The differences were considerable (*P* < 0.05).

### 3.2. Prognostic Risk Factors of HBV-Associated ACLF Patients

Table 1 shows the single-factor and multifactor logistic regression analysis. In the univariate analysis of the prognosis of HBV-associated ACLF patients, TBIL (*P*=0.004), PT (*P*=0.012), APTT (*P*=0.005), and IL-26 (*P* < 0.001) were considerable. In the multivariate analysis, TBIL (*P*=0.035) and IL-26 (*P*=0.013) were independent predictors of the prognosis of patients with HBV-associated ACLF.

### 3.3. Analysis of CT Image Low-Density Foci Segmentation Results Based on Three Algorithms

In Figure 6, the machine learning-based algorithms Deep Medic and Seg Net were compared with the 3D-CNN model. According to the Dice coefficient of the segmentation results, the Dice coefficient of 3D-CNN (0.884 ± 0.068) in the overall segmentation of low-density stoves was slightly lower than Deep Medic algorithm (0.900 ± 0.077) and higher than Seg Net algorithm (0.846 ± 0.072). In the core segmentation of low-density foci, the Dice coefficient of 3D-CNN was 0.821 ± 0.07, which was higher than Deep Medic algorithm (0.763 ± 0.069) and Seg Net algorithm (0.754 ± 0.076). In the segmentation of enhanced lesions, the Dice coefficient of 3D-CNN (0.773 ± 0.071) was higher than that of Deep Medic algorithm (0.731 ± 0.074) and Seg Net algorithm (0.694 ± 0.078), and the difference was considerable (*P* < 0.05).

A 53-year-old male patient presented with intermittent abdominal distension for two years with exacerbation and yellowing of eyes and skin for two weeks. CT examination two years ago showed cirrhosis. That time, the patient visited the hospital due to abdominal distension and fatigue. HBsAg (+), HBeAg (−), and HBV DNA 2.46 × 10^5^ IU/mL were examined.  Figure 7 shows the results of segmentation of low-density foci by different algorithm models. Green was the lesion area marked by the doctor, and red was the lesion area automatically marked by the three algorithm models. The 3D-CNN marked the area more closely to the area the doctor had sketched by hand.

### 3.4. Comparison of CT Image Candidate Detection Results Based on Three Algorithms

The results of candidate detection of nodular lesions using different algorithms are shown in Figure 8. The number of nodular lesions detected by 3D-CNN was 533, which was higher than that of Deep Medic algorithm (506) and Seg Net algorithm (482). Sensitivity (97.5%) of 3D-CNN was higher than that of Deep Medic algorithm (95.6%) and Seg Net algorithm (93.8%). The missed detection rate (0.52%) of 3D-CNN was lower than that of Deep Medic algorithm (0.76%) and the Seg Net algorithm (1.25%), and the difference was considerable (*P* < 0.05).

## 4. Discussion

HBV-associated ACLF is a reaction after a series of injuries, such as systemic immune disorders due to various inducements of acute liver injury based on chronic liver disease [21, 22]. It causes severe liver damage or failure. HBV-ACLF can lead to rapid deterioration of liver function, circulatory system, and organ dysfunction in the course of disease development, which is of high mortality and poor prognosis [23]. Many studies deemed that immune dysfunction is the main cause of ACLF. In the early stage, immune overexcitation and continuous inflammatory response cause a large number of liver cell necrosis [24, 25], while inflammatory cell infiltration and microcirculation disorder also exist. With the progress of the disease, liver failure, toxin accumulation in the body, internal environment disorder, and other consequences gradually appear [26]. In clinical practice, experts usually segment lesions manually based on their professional knowledge and work experience. The method based on computer automatic segmentation can effectively help doctors relieve working pressure and quickly and accurately obtain the feedback of the lesion area to doctors [27], which provides good diagnostic conditions and recommendations for treatment options. In clinical practice, CNN is usually used to build a medical image segmentation algorithm model to assist physicians to greatly improve the analysis effect of imaging features [28]. In this study, liver function and serum inflammatory cytokine levels were detected in 30 HBV-ACLF patients, 30 CHB patients, and 30 healthy volunteers. The end-to-end neural network architecture based on 3D-CNN was designed and applied to CT image analysis.

The results showed that the levels of IL-6, IL-26, and IL-37 were the highest in HBV-ACLF group, and TBIL and IL-26 were independent predictors of the prognosis of HBV-ACLF patients. The results of focal segmentation showed that the Dice coefficient of low-density focal core and enhanced focal segmentation was the highest in 3D CNN, and the labeled regions were closer to the regions delineated manually by doctors. Moreover, 3D CNN was superior to other algorithms in the number, sensitivity, and missed detection rate of nodular lesions detected (*P* < 0.05). In short, IL-26 may be a useful biomarker in the treatment of HBV-ACLF. The 3D-CNN model improved the segmentation performance of lesions in CT images of patients with HBV-ACLF, providing a reference for the diagnosis and prognosis of HBV-ACLF. This is consistent with the research results of Osuna-Coutiño and Martinez-Carranza [29]. 3D-CNN model makes full use of the interlayer information of CT images to improve the continuity of CT image segmentation. Hamidian et al. [30] pointed out that 3D-CNN combined the advantages of 2D and 3D models and significantly improved the segmentation performance of the model. It was found that TBIL and IL-26 were independent predictors of prognosis in patients with HBV-ACLF, and IL-26 may be a useful biomarker in the treatment of HBV-ACLF.

## 5. Conclusion

In this study, an intelligent CT image segmentation model based on 3D-CNN algorithm was established to integrate 2D and 3D models, which was applied to CT images of HBV-ACLF patients. The results showed that the 3D-CNN algorithm model had ideal performance in CT image segmentation of HBV-ACLF patients. However, there are still some shortcomings in this study. The experimental results have certain limitations and one-sidedness, so it is necessary to increase the sample size in the future and conduct further exploration in this direction. In conclusion, 3D-CNN model greatly improves the segmentation performance of CT images of patients with HBV-ACLF, which provides a reference for the diagnosis and prognosis of HBV-ACLF.

## Figures and Tables

**Figure 1:** Structure diagram of CNN.

**Figure 2:** Local connection and weight sharing.

**Figure 3:** Basic network structures of 3D-CNN.

**Figure 4:** 3D-CNN's low-density foci segmentation process.

**Figure 5:** Comparison of the levels of inflammatory factors among the three groups of objects. Note: ^*∗*^ indicates that the level of inflammatory factors in the HBV-ACLF group had a considerable difference compared with the CHB group and the HC group (*P* < 0.05).

**Figure 6:** Analysis of CT image low-density lesion segmentation results based on three algorithms. Note: ^*∗*^ indicates that the Dice coefficient of the 3D-CNN model was considerable compared to the other two algorithms (*P* < 0.05).

**Figure 7:** Different algorithm models segmentation results of low-density foci. (a) The CT image marked by the Deep Medic algorithm model, (b) the CT image marked by the Seg Net algorithm model, and (c) the CT image marked by the 3D-CNN model.

**Figure 8:** Comparison of CT image candidate detection results based on three algorithms. (a) The comparison of the number of nodular lesions detected by the three algorithms. (b) The comparison of the sensitivity and missed detection rate of the three algorithms. Note: ^*∗*^indicates that the detection performance of the 3D-CNN model was considerable compared to the other two algorithms (*P* < 0.05).

**Table 1:** Prognostic risk factors of HBV-associated ACLF patients.

	*P*	Univariate analysis OR	95% CI	*P*	Multifactor analysis OR	95% CI
ALT (U/L)	0.291	1.000	0.987–1.000			
AST (U/L)	0.698	1.000	0.995–1.000			
TBIL (*μ*mol/L)	0.004	1.0078	1.004–1.021	0.035	1.015	1.000–1.026
PT (s)	0.012	1.136	1.031–1.215	0.388	1.356	0.682–2.521
APTT (s)	0.005	1.043	1.008–1.098	0.891	1.002	0.936–1.054
IL-6 (pg/mL)	0.077	1.253	0.998–1.561	0.605	0.187	0.001–1.298
IL-26 (pg/mL)	≤0.001	1.004	0.936–1.006	0.013	1.005	1.000–1.006
IL-37 (pg/mL)	0.340	0.991	0.972–1.008	0.072	1.015	0.993–1.066

## Data Availability

The data used to support the findings of this study are available from the corresponding author upon request.

## References

[1] Solé C., Solà E. (2018). Update on acute-on-chronic liver failure. *Gastroenterología Y Hepatología (English Edition)*.

[2] Gustot T., Jalan R. (2019). Acute-on-chronic liver failure in patients with alcohol-related liver disease. *Journal of Hepatology*.

[3] Wu D., Zhang S., Xie Z. (2020). Plasminogen as a prognostic biomarker for HBV-related acute-on-chronic liver failure. *Journal of Clinical Investigation*.

[4] Li C., Su H.-B., Liu X.-Y., Hu J.-H. (2020). Clinical characteristics and 28-d outcomes of bacterial infections in patients with hepatitis B virus-related acute-on-chronic liver failure. *World Journal of Clinical Cases*.

[5] Liu H., Zhang Q., Liu L. (2020). Effect of artificial liver support system on short‐term prognosis of patients with hepatitis B virus‐related acute‐on‐chronic liver failure. *Artificial Organs*.

[6] Jia Y., Ma L., Wang Y. (2020). NLRP3 inflammasome and related cytokines reflect the immune status of patients with HBV-ACLF. *Molecular Immunology*.

[7] Shen G., Sun S., Huang J. (2020). Dynamic changes of T cell receptor repertoires in patients with hepatitis B virus-related acute-on-chronic liver failure. *Hepatology International*.

[8] Schmid E., Leeson K., Xu K. T., Richman P., Nwosu C., Carrasco L. (2019). CT imaging history for patients presenting to the ED with renal colic--evidence from a multi-hospital database. *BMC Emergency Medicine*.

[9] Matthews M., Richman P., Krall S. (2018). Prior CT imaging history for patients who undergo whole-body CT for acute traumatic injury and are discharged home from the emergency department. *BMC Emergency Medicine*.

[10] Jha S. (2019). Coronary computed tomography. *PET Clinics*.

[11] Desai V., Cox M., Deshmukh S., Roth C. G. (2018). Contrast-enhanced or noncontrast CT for renal colic: utilizing urinalysis and patient history of urolithiasis to decide. *Emergency Radiology*.

[12] Fukukura Y., Kumagae Y., Higashi R. (2020). Visual enhancement pattern during the delayed phase of enhanced CT as an independent prognostic factor in stage IV pancreatic ductal adenocarcinoma. *Pancreatology*.

[13] Willemink M. J., Noël P. B. (2019). The evolution of image reconstruction for CT-from filtered back projection to artificial intelligence. *European Radiology*.

[14] Kambadakone A. (2020). Artificial Intelligence and CT image reconstruction: potential of a new era in radiation dose reduction. *Journal of the American College of Radiology*.

[15] Yang X., Wang N., Song B., Gao X. (2019). BoSR: a CNN-based aurora image retrieval method. *Neural Networks*.

[16] Hsieh T.-H., Kiang J.-F. (2020). Comparison of CNN algorithms on hyperspectral image classification in agricultural lands. *Sensors*.

[17] Feng F., Wang S., Wang C., Zhang J. (2019). Learning deep hierarchical spatial-spectral features for hyperspectral image classification based on residual 3D-2D CNN. *Sensors*.

[18] Yu J., Yang B., Wang J., Leader J., Wilson D., Pu J. (2020). 2D CNN versus 3D CNN for false-positive reduction in lung cancer screening. *Journal of Medical Imaging*.

[19] Sarin S. K., Choudhury A., Choudhury A. (2019). Acute-on-chronic liver failure: consensus recommendations of the Asian Pacific association for the study of the liver (APASL): an update. *Hepatology International*.

[20] Chinese Society of Hepatology (2005). Chinese medical association; Chinese society of infectious diseases, Chinese medical association. [the guidelines of prevention and treatment for chronic hepatitis B]. *Zhonghua Gan Zang Bing Za Zhi*.

[21] Sun Z., Liu X., Wu D. (2019). Circulating proteomic panels for diagnosis and risk stratification of acute-on-chronic liver failure in patients with viral hepatitis B. *Theranostics*.

[22] Yao J., Li S., Zhou L. (2019). Therapeutic effect of double plasma molecular adsorption system and sequential half‐dose plasma exchange in patients with HBV‐related acute‐on‐chronic liver failure. *Journal of Clinical Apheresis*.

[23] Pang X., Li X., Mo Z. (2018). IFI16 is involved in HBV-associated acute-on-chronic liver failure inflammation. *BMC Gastroenterology*.

[24] Yan Q., Wang L., Lai L. (2019). Next generation sequencing reveals novel alterations in B-cell heavy chain receptor repertoires associated with acute-on-chronic liver failure. *International Journal of Molecular Medicine*.

[25] Liu F., Duan X., Wan Z. (2016). Lower number and decreased function of natural killer cells in hepatitis B virus related acute-on-chronic liver failure. *Clinics and Research in Hepatology and Gastroenterology*.

[26] Zhang D.-N., Liu Y., Li X. (2021). Imbalance between soluble and membrane-bound CD100 regulates monocytes activity in hepatitis B virus-associated acute-on-chronic liver failure. *Viral Immunology*.

[27] Dong X., Lei Y., Wang T. (2019). Automatic multiorgan segmentation in thoraxCTimages using U‐net‐GAN. *Medical Physics*.

[28] Zhou X. (2020). Automatic segmentation of multiple organs on 3D CT images by using deep learning approaches. *Advances in Experimental Medicine and Biology*.

[29] Osuna-Coutiño J., Martinez-Carranza J. (2019). High level 3D structure extraction from a single image using a CNN-based approach. *Sensors*.

[30] Hamidian S., Sahiner B., Petrick N., Pezeshk A. (2017). 3D convolutional neural network for automatic detection of lung nodules in chest CT. *Medical Imaging 2017: Computer-Aided Diagnosis*.

